The article "Effect of Electroacupuncture on Noise-Induced Hearing Loss in Rats" was published in 2021. Journal: Evid Based Complement Alternat Med.

# Effect of Electroacupuncture on Noise-Induced Hearing Loss in Rats

**DOI:** 10.1155/2021/9114676

**Published:** 2021-10-27

**Authors:** Chia-Hao Chang, Chia-Der Lin, Ching-Liang Hsieh

**Affiliations:** ^1^Graduate Institute of Acupuncture Science, China Medical University, Taichung, Taiwan; ^2^Department of Chinese Medicine, China Medical University Hospital, Taichung, Taiwan; ^3^Division of Otorhinolaryngology, China Medical University Hospital, Taipei Branch, Taiwan; ^4^Department of Otorhinolaryngology, China Medical University Hospital, Taichung, Taiwan; ^5^School of Medicine, China Medical University, Taichung, Taiwan; ^6^Chinese Medicine Research Center, China Medical University, Taichung, Taiwan

## Abstract

Acupuncture has long been used to relieve some inner ear diseases such as deafness and tinnitus. The present study examined the effect of electroacupuncture (EA) on noise-induced hearing loss (NIHL) in animals. A NIHL rat model was established. Electroacupuncture pretreatment at 2 Hz or posttreatment at the right Zhongzhu (TE3) acupoint was applied for 1 hour. Auditory thresholds were measured using auditory brainstem responses (ABRs), and histopathology of the cochlea was examined. The results indicated that the baseline auditory threshold of ABR was not significantly different between the control (no noise), EA-only (only EA without noise), noise (noise exposure only), pre-EA (pretreating EA then noise), and post-EA (noise exposure then posttreating with EA) groups. Significant auditory threshold shifts were found in the noise, pre-EA, and post-EA groups in the immediate period after noise exposure, whereas auditory recovery was better in the pre-EA and post-EA groups than that in the noise group at the three days, one week (W1), two weeks (W2), three weeks (W3), and four weeks(W4) after noise stimulation. Histopathological examination revealed greater loss of the density of spiral ganglion neurons in the noise group than in the control group at W1 and W2. Although significant loss of spiral ganglion loss happened in pre-EA and post-EA groups, such loss was less than the loss of the noise group, especially W1. These results indicate that either pretreatment or posttreatment with EA may facilitate auditory recovery after NIHL. The detailed mechanism through which EA alleviates NIHL requires further study.

## 1. Introduction

Noise-induced hearing loss (NIHL) is the second most common cause of acquired hearing loss, and NIHL is defined as sensorineural deafness due to long- or short-term noise exposure [1]. NIHL is often caused by long-term occupational exposure to noise [2]. The prevalence of hearing loss due to noise varies from 11.2% to 58% globally [3]. Hearing impairment can cause communication difficulty, social isolation, emotional depression, and cognitive decline, which can result in health problems, increase hospitalization, affect quality of life, and increase the burden on the family and society [4]. Therefore, avoiding NIHL and developing an effective treatment strategy are important.

The article "Effect of Electroacupuncture on Noise-Induced Hearing Loss in Rats" was published in 2021. Journal: Evid Based Complement Alternat Med.

Exposure to intense auditory stimulation may induce a temporary threshold shift or permanent threshold shift. There are many studies to investigate the molecular mechanism of NIHL, including the accumulation of reactive oxygen species (ROS) and the activation of the intracellular stress signal pathway, which results in programmed or necrotic cell death and, eventually, the permanent damage of cochlear hair cells and synapses, leading to the development of NIHL [5]. The physical mechanisms of NIHL include physical damage of the organ of Corti; a reduction in blood flow in the inner ear; the accumulation of free radicals, such as ROS; and the degeneration of cochlear nerve fibers in synaptic terminals and spiral ganglion neurons [6].

High doses of steroids with or without hyperbaric oxygen treatment might be effective for acute NIHL [7]. Several other drugs have been investigated experimentally for the treatment of NIHL, such as glutamate inhibitors (caroverine), anti-ischemic agents (trimetazidine dihydrochloride), and antioxidants (glutathione) [8, 9]. However, these agents are still controversial or limited in real clinical application. Caroverine would have the side effects of headache, nausea, and dizziness. The reports about the effectiveness of trimetazidine dihydrochloride in treating NIHL are controversial [10]. The study of antioxidants is only limited in the animal model study. Hyperbaric oxygen therapy is expensive, time-consuming with controversial results. Steroids, though may be effective, would produce some long-term side effects in human beings. Therefore, acupuncture or electroacupuncture (EA) has its traditional role in treating some inner ear problems such as tinnitus or hearing loss, but direct evidence is still lacking to prove its role. The purpose of this study is to investigate the effect of EA in NIHL in animals.

In traditional Chinese medicine (TCM), the Zhongzhu (TE3) acupoint is located on the triple energizer meridian of the hand that is connected to the ear. Acupuncture at TE3 exerts beneficial effects on auditory function, and it can treat deafness and tinnitus [11]. A functional magnetic resonance imaging study showed that acupuncture at bilateral TE3 causes the excitation of bilateral acoustic, occipital, and sensorimotor cortices [12]. Electroacupuncture (EA) at the periauricular acupoints and adjuvant TE3 restores refractory unilateral sensorineural hearing loss [13]. A randomized, parallel, open-labeled trial shows that EA at distal acupoints including TE3 has a similar effect to EA at periauricular acupoints in improving tinnitus [14]. Acupuncture at distal acupoints TE3 can ameliorate tinnitus in patient with the improvement of cochlear blood flow [15]. However, there are still lacking direct evidence to verify the role of EA in inner ear disorders such as NIHL in animals. Holt et al. report that the Sprague Dawley (SD) rat noise injury model can tolerate exposure to loud sounds, long-term effect study, and also can provide the information of the morphology, nervous system function, and neuronal activity for preclinical study [16]. Therefore, the present study investigated the prevention and the treatment effect of EA at TE3 on hearing loss in SD rats with NIHL.

The article "Effect of Electroacupuncture on Noise-Induced Hearing Loss in Rats" was published in 2021. Journal: Evid Based Complement Alternat Med.

## 2. Materials and Methods

### 2.1. Animals

Male SD rats, aged from 8 to 12 weeks, were purchased from BioLASCO Taiwan and were reared in the Animal Center of China Medical University. The rats were placed together in a cage in a regular light and dark environment (12/12 hours); an air conditioner was used to maintain the room temperature at 22–24°C and the humidity at 50%–70%. The rats were provided with adequate food and water ad libitum. All experimental procedures were performed in accordance with the guidelines of the Animal Experimental Ethics Committee (IACUC-2016-120).

### 2.2. Noise-Induced Hearing Loss Model

The animals were sedated by intraperitoneal injection of Zoletil (20 mg/kg) and Xylazine (5 mg/kg) and then maintenance with Zoletil (10 mg/kg) and Xylazine (2.5 mg/kg) when necessary. Broadband white noise (1–20 kHz) stimulation at the intensity of 121 dB was administered to the animals in a sound-proof box for 2 hours after the animals were sedated. The noise spectrum and dose were determined according to our pilot study, and the report of Park et al. was referred [17]. Subsequently, auditory brainstem responses (ABR) were used to assess their hearing.

### 2.3. ABR Recording

The auditory threshold was assessed using ABR, as described in our previous research [18]. In brief, first, the earphone was inserted into the external auditory canal of the rat; a subcutaneous needle electrode was then placed high on their forehead as a reference electrode, and the other subcutaneous needle electrode was placed on the mastoid as a recording electrode. Another subcutaneous needle electrode was placed low on the forehead as a ground electrode. These electrodes were connected to an auditory evoked potential system (SmartEP, Intelligent Hearing System, 6860 SW 81st St, Miami, FL 33143, USA).

The article "Effect of Electroacupuncture on Noise-Induced Hearing Loss in Rats" was published in 2021. Journal: Evid Based Complement Alternat Med.

ABR recording was performed in which a tone burst was generated from the auditory evoked potential system in a soundproof room. The ABR sound is emitted by the processing system with the following parameters: a rise/fall period of 0.5 ms, stimulus duration of 1 ms, and sweep of 1024 times at a rate of 19.30/s. The sound stimulation comprised clicks, with a tone burst at 2, 4, and 8 kHz. ABRs were obtained at each frequency by reducing the sound pressure level in 10 dB steps from a maximum of 80 dB to a minimum of 0 dB at which the ABR response disappeared. The threshold was defined as the lowest level at which an ABR wave could be recognized. The threshold shift (dB) was obtained by subtracting the hearing threshold after the intervention and the hearing threshold before the intervention.

### 2.4. Experimental Grouping

The present study was divided into experiments A and B.

#### 2.4.1. Experiment A Investigated the Effect of EA on Hearing Recovery Time in Rats with NIHL

The animals were divided into five groups (*n* = 7 per group) as follows: (1) control group, animals without noise exposure or other treatment; (2) EA-only group, animals receiving EA treatment only without NIHL; (3) noise group, animals receiving noise exposure as previously described and without other treatment; (4) pre-EA group, animals pretreated with EA prior to noise exposure as previously described (i.e., Pre-EA + noise); and (5) post-EA group, animals receiving EA treatment immediate after noise exposure (i.e., noise + post-EA).

Baseline auditory level was recorded with ABR before noise exposure or EA treatment. Subsequently, ABR recording was conducted immediately (Im), 3 days (D3), 1 week (W1), 2 weeks (W2), 3 weeks (W3), and 4 weeks (W4) after noise stimulation. Finally, the rats were sacrificed after 4 weeks of ABR recording. The experimental procedure is summarized in Figure 1.

#### 2.4.2. Experiment B Histopathological Investigation of the Effect of EA in Rats with/without NIHL

According to the results in experiment A, histopathological examination, especially spiral ganglion neuron, was investigated. A total of 34 rats were studied, and the rats were divided into five groups (as in Experiment A), with 4 rats in each group except for 2 rats in the control group.

### 2.5. EA Treatment

First, the rats were anesthetized as described above; then, a stainless-steel acupuncture needle (2.54 cm in length, 34 No., Hian Huei Acupuncture Appliance, Taiwan) was inserted into the right Zhongzhu point (TE3), which is comparable to the location on the dorsum of the hand between the fourth and fifth metacarpal bones in humans. Another needle was inserted 0.5 cm proximal to TE3; then, the needles were connected to an electrostimulation apparatus (Trio 300, Japan). The parameters of EA treatment in this study were as follows: frequency of 2 Hz, width of 250 *μ*s, intensity of 2 mA, and duration of 1 hour [19].

The article "Effect of Electroacupuncture on Noise-Induced Hearing Loss in Rats" was published in 2021. Journal: Evid Based Complement Alternat Med.

### 2.6. Histopathological Examination

The rats were sacrificed at W1 and W2 after click stimulation; then, left cochlear sectioning was performed along the paramodiolar axis, followed by hematoxylin/eosin staining. After the aforementioned fixation procedure was executed, the cochleae were decalcified in 10% ethylene-diamine tetra-acetic acid (EDTA) for 4 weeks at 4°C, dehydrated, embedded in paraffin, and sectioned serially (4 *μ*m thick) parallel to the modiolar axis [20]. The specimens were observed with the spiral ganglion cells counted under a light microscope (Olympus BX51) and photographed (Olympus U-25ND6), and the digital images were saved. After the image collected, we used ImageJ software to encircle the exterior of spiral ganglion cells, then calculate the density of spiral ganglion cells by defining control group as 100%, and then calculate it for other groups proportionally.

### 2.7. Statistical Analysis

The auditory threshold shifts among the control, EA, noise, pre-EA, and post-EA groups were analyzed using one-way ANOVA with Tukey's honestly significant difference (HSD) post hoc test. Then, we used repeated measurement ANOVA with a Greenhouse–Geisser correction to determine the mean auditory threshold shift among different treatment groups across 6 time points of Im, D3, W1, W2, W3, and W4. The percentages of spiral ganglion neurons and histopathological examination results of the control, EA-only, noise, pre-EA, and post-EA groups were analyzed using one-way ANOVA with Tukey's HSD. Statistical significance was indicated if *p* < 0.05.

## 3. Results

### 3.1. Experiment A

#### 3.1.1. Effect of EA on Auditory Threshold Shifts in Rats with/without NIHL

In the measurement of ABR threshold using the click stimulation, the baseline (before noise exposure) auditory threshold of ABR was similar among the control, EA-only, noise, pre-EA, and post-EA groups (all *p* > 0.05). Immediately after noise exposure, significant auditory threshold shifts were observed in the noise, pre-EA, and post-EA group, though there no significant difference among these groups. No significant auditory threshold shifts were observed in the control and EA-only groups from baseline, Im, D3, W1, W2, W3, to W4. Significant recovery of auditory threshold shifts was observed in the pre-EA and post-EA groups at D3, W1, W2, W3, and W4 after noise stimulation, compared with that in the noise group. The auditory recovery in the both pre-EA and post-EA group started from D3 and gradually got recovered near the auditory level of control or the EA-only group at W3 and W4. All *p* values for all pairs of the aforementioned groups are shown in Figure 2.

The article "Effect of Electroacupuncture on Noise-Induced Hearing Loss in Rats" was published in 2021. Journal: Evid Based Complement Alternat Med.

In the measurement of ABR threshold shifts using 2 kHz, 4 kHz, and 8 kHz tone burst stimulation, the results are similar to those using click stimulation. All *p* values between all pairs of the aforementioned groups are shown in Figure 2.

### 3.2. Experiment B

#### 3.2.1. Effect of EA at TE3 on Spiral Ganglion Cells in Rats with NIHL

The density of spiral ganglion neurons was similar between the control and EA-only groups in W1 and W2. The density of spiral ganglion neurons was similar among the pre-EA, post-EA, and EA only groups in W1. Compared with the control group, significant loss of spiral ganglion neurons was observed in the noise and post-EA groups (*p* < 0.0001 and *p* < 0.05, respectively; Figures 3(a) and 3(b)). Compared with the spiral ganglion neurons in the noise group, less loss of spiral ganglion neurons was observed when the animals were pretreated with EA in W1 (*p* < 0.001; Figures 3(a) and 3(b)). The density of spiral ganglion neurons was similar between the control and EA-only groups (*p* > 0.05; Figures 3(a) and 3(b)) at W2. The density of spiral ganglion neurons was greater in the control group than in the noise, pre-EA, and post-EA groups in W2 (*p* < 0.0001, *p* < 0.01, and *p* < 0.001, respectively; Figures 3(a) and 3(b)); the density of spiral ganglion neurons was greater in the EA-only group than in the noise and post-EA groups (*p* < 0.01 and *p* < 0.05, respectively; Figures 3(a) and 3(b)); the density of spiral ganglion neurons was greater in the pre-EA group than in the noise group (*p* < 0.05; Figures 3(a) and 3(b)).

## 4. Discussion

The results of the present study indicated that the auditory threshold of ABR was similar in the five groups (control, EA-only, noise, pre-EA, and post-EA groups) before noise stimulation (baseline period), whereas in the immediate period after noise exposure, the auditory threshold shifts of ABR in the noise, pre-EA, and post-EA groups were more significant than those in the control and EA-only groups. These results indicated that NIHL was successfully induced in the rats in the present study because the control and EA-only groups did not receive noise stimulation. In addition, EA only does not exert adverse effects on auditory function. The recovery of auditory threshold shifts in the pre-EA and post-EA groups were better than those in the noise group. Eventually, the recovery of auditory threshold shifts in the pre-EA and post-EA groups was near the hearing levels of control and EA-only groups at 3-4weeks after noise exposure. The hearing threshold shift of ABR was similar in the control, EA-only, pre-EA, and post-EA groups at W3 and W4.

The article "Effect of Electroacupuncture on Noise-Induced Hearing Loss in Rats" was published in 2021. Journal: Evid Based Complement Alternat Med.

Histopathological examination showed that the density of spiral ganglion neurons in the noise group was significantly lower than that in the control group at W1 and W2 and was also lower than that in the EA-only group at W2. This indicated that our NIHL model is successful to damage to the spiral ganglion neurons occurred after noise exposure significantly. In W1 and W2, such spiral ganglion neuron density between noise and pre-EA had significant difference (*p* < 0.001 and *p* < 0.05, respectively). This indicated that the spiral ganglion might be recovered by pretreatment with EA. These results suggest that EA may recover hearing ability damaged from noise injury and that EA pretreatment may also exert a protective effect in rats from noise trauma. This result is also consistent with the theory of TCM, EA at TE3 induces the generation of qi, and that along the triple energizer meridian reach to inner ear produces protective effect for inner ear disorders, such as NIHL [11].

NIHL is caused by the transmission of intense noise energy to the inner ear, resulting in the mechanical damage of hair cells, disruption of synapses, production of oxidative stress, damage of the biological membrane, influx of Ca^2+^ into hair cells, and development of immune and inflammatory reactions in the inner ear [1, 6]; furthermore, noise induces the reduction of blood flow, resulting in the hypoxia of the inner ear [6]. TE3 is located on the triple energizer meridian of the hand that is connected to the ear according to the acupuncture guidelines for selecting acupoints (“where the meridian passes, “that point” can be used for the treatment of diseases”) [11]. Therefore, EA at TE3 often is applied to treat inner ear diseases, such as deafness and tinnitus.

The precise mechanism of acupuncture is still not clear. There might be various mechanisms in different applications. Acupuncture can increase cerebral blood flow in patients with stroke [21] and in rats with multiple infarction dementia [22]. EA at Zusanli (ST36) and Sanyinjiao (SP6) exerts neuroprotective effects in a mouse model of Parkinson's disease through antioxidant and antiapoptotic effects [23]. The anti-inflammatory action of acupuncture plays a crucial role in acupuncture analgesia, especially for inflammatory pain [24], and electric stimulation at the ear and EA at ST36–ST37 can reduce the number of cyclooxygenase-2 (COX2) immunoreactive cells in the CA1 region of the hippocampus; thus, these therapies exert anti-inflammatory effects in kainic acid-induced epileptic rats [25]. Acupuncture can play an immunomodulatory role in the immune system through the activation of macrophages and the complementary system and the generation of immunoglobulins [26]. EA applied to ST36 can maintain the intestinal mucosal immune barrier by increasing the number of CD3+ T cells and the ratio of CD4+/CD8+ T cells in rats with sepsis induced by cecal ligation and puncture [27]. In the present study, the findings indicated that pretreatment or posttreatment with 2-Hz EA at the right TE3 enhanced the auditory threshold shift recovery of ABR, possibly through multiple pathways, including increased blood flow of the inner ear, antioxidant effects, and anti-inflammatory effects. In addition, EA possibly induces the effect of neurotransmitters including opioids peptides and glutamates and also activates calcium ion channels, and these effects change neural signaling transmission [13, 28], but the real mechanism remains unclear and requires further study.

The article "Effect of Electroacupuncture on Noise-Induced Hearing Loss in Rats" was published in 2021. Journal: Evid Based Complement Alternat Med.

The present study results indicated that the auditory threshold shift of ABR was similar in the pre-EA and post-EA groups at Im, D3, W1, W2, W3, and W4 in the click and 2, 4, and 8 KHz tone burst stimulation. However, the preservation of spiral ganglion neurons was significantly better in the pre-EA group than that in the noise group, but the post-EA group did not show such significant different with the noise group. The findings suggest EA pretreatment might play a preventive effect for spiral ganglion neurons in the rats with NIHL, but the effect in the EA posttreatment is not obvious. This result is consistent with a good doctor who starts treatment before the onset of the disease, if the treatment after the onset of the disease is too late that is mentioned in the book of “Yellow Emperor's Canon of Internal Medicine” [29].

Some questions remain that require further study, for example, why EA applied at the right TE3 can improve the auditory threshold shift of ABR of the left ear? According to TCM guidelines, the circulation of meridian qi is like a ring with no end [29], and if the disease is on the left, the treatment can be acupuncture on the right side, and if the disease is on the right, the treatment can be acupuncture on the left side [29]. Fascia is integrated with mutual influence because both sides of the fascia are connected. Treatment applied to the right side also affects the left side [30]. Our previous study shows EA at contralesioned scalp can increase gamma-aminobutyric acid (GABA) A levels of lesioned hemisphere and reduces infarction volume in rats with ischemia-reperfusion injury [31], and EA at contralateral ST36 and GB34 can prolong first demand time of patient-controlled analgesia (PCA) in patients with total knee arthroplasty [32]. However, the underlying mechanisms should be explored in the future. In the present study, EA was applied to TE3 for 1 hour and only once, which was similar to an animal study showing EA with lower frequency (3 Hz) and longer duration (60 minutes) would increase nociceptive thresholds and persist for longer period [19]. In the present study, we established an EA-only group to prove the EA therapy is no harm to hearing ability, but lacks a sham EA group to better prove the efficacy of EA. Therefore, the study was preliminary, and a sham EA group will be designed in the future.

The article "Effect of Electroacupuncture on Noise-Induced Hearing Loss in Rats" was published in 2021. Journal: Evid Based Complement Alternat Med.

In conclusion, noise stimulation can induce the auditory threshold shift of ABR, and this shift was improved in the pre-EA and post-EA groups. In addition, the density of spiral ganglion neurons was increased in the pre-EA group, suggesting that 2-Hz EA at right TE3 (pretreatment or posttreatment) is helpful for auditory recovery in rats with noise exposure, and EA pretreatment also has protective effects on spiral ganglion neurons.

## Figures and Tables

**Figure 1:** In total, 35 rats were divided into five groups (7 rats in the group for experiment A). Control: the control group did not receive 121-dB noise stimulation or electroacupuncture (EA) treatment; pre-EA: pre-EA group received 2-Hz EA treatment at TE3 (intensity of 2 mA for 1 hour) prior to noise stimulation; noise: the noise group received 121-dB noise stimulation for 2 hours only; post-EA: post-EA group received EA treatment at TE3 after noise stimulation; EA-only: EA-only group received EA treatment at TE3 only. ABR: auditory brain stem response; baseline: ABR recording prior to EA or noise treatment; Im.: immediate period after noise stimulation; day 3 (D3): 3 days after noise stimulation; week 1 (W1): 1 week after noise stimulation; week 2 (W2): 2 weeks after noise stimulation; week 3 (W3): 3 weeks after noise stimulation; week 4 (W4): 4 weeks after noise stimulation; yes: performed; no: not performed.

**Figure 2:** Effect of electroacupuncture at right TE3 on auditory threshold shift of auditory brain stem response in rats with noise-induced hearing loss. Auditory threshold shift of the auditory brain stem response was observed in the noise, pre-EA, and post-EA groups in the immediate period after noise stimulation, whereas this shift was greatly reduced in the pre-EA and post-EA group at D3, W1, W2, W3, and W4. No prominent auditory threshold shift was found in the control and EA-only groups. At W3 and W4, the auditory threshold shift was similar in the control, EA-only, pre-EA, and post-EA groups in the click and 2, 4, and 8 KHz tone burst stimulation. ^★★^*p* < 0.01, ^★★★^*p* < 0.001 control vs. noise; ^◆^*p* < 0.05, ^◆◆^*p* < 0.01, ^◆◆◆^*p* < 0.001 control vs. post-EA; ^†^*p* < 0.05, ^††^*p* < 0.01, ^†††^*p* < 0.001 control vs. pre-EA; ^●^*p* < 0.05, ^●●^*p* < 0.01, ^●●●^*p* < 0.001 noise vs. pre-EA; ^◇^*p* < 0.05, ^◇◇^*p* < 0.01, ^◇◇◇^*p* < 0.001 noise vs. post-EA; ^Δ^*p* < 0.05 pre-EA vs. post-EA.

The article "Effect of Electroacupuncture on Noise-Induced Hearing Loss in Rats" was published in 2021. Journal: Evid Based Complement Alternat Med.

**Figure 3:** Effect of electroacupuncture at right TE3 on spiral ganglion neurons in rats with noise-induced hearing loss. The density of spiral ganglion neurons (arrow head) was greater in the control group (control) than in the noise group (noise); EA pretreatment at right TE3 increased the density of spiral ganglion neurons. pre-EA: pre-EA group; post-EA: post-EA group; EA: EA-only group; (a) Density of spiral ganglion neurons. (b) Statistical analysis chart; W1: 1 week after noise stimulation; W2: 2 weeks after noise stimulation;  ^*∗∗*^*p* < 0.01, ^*∗∗*^*p* < 0.01,  ^*∗∗∗*^*p* < 0.001, and  ^*∗∗∗∗*^*p* < 0.0001.

## Data Availability

The data in this study are available to other researchers upon request.
